RETRACTED

# Exploring the Independent Learning of Music Students in Higher Teacher Training Colleges in a Pluralistic Network Environment

**DOI:** 10.1155/2022/5024006

**Published:** 2022-06-28

**Authors:** Lei Zhang

**Affiliations:** Department of Music, Tangshan Normal University, Tangshan 063000, China

## Abstract

As the main base for training teachers, normal colleges and universities can not only reserve a large number of talents for the construction of teachers but also help to improve the professional quality and teaching ability of teachers. Carrying out research on music education in normal colleges and universities can further meet the diversified needs of the current society for music talents and promote the improvement of art cultivation and cultural level of music students in normal colleges and universities. This paper discusses the preparation work of higher normal music colleges under the new curriculum standards from four aspects: “experience learning, independent learning, cooperative learning, and inquiry learning.” Later, through the method of questionnaire survey, starting from the survey of the independent learning motivation of 325 music education students, the independent learning situation of music education students under the network resources was analyzed, and the learning strategies were discussed from various aspects of students, teachers, and the school. By analyzing the current situation of music teaching in higher teacher training colleges from many aspects, and putting forward relevant suggestions according to the survey results, we hope to help the transformation of music teaching methods in the future and make contributions to the field of music teaching in China.

## 1. Introduction

As the main base for training teachers, normal colleges and universities can not only reserve a large number of talents for the construction of teachers but also help to improve the professional quality and teaching ability of teachers. Carrying out research on music education in normal colleges and universities can further meet the diversified needs of the current society for music talents and promote the improvement of art cultivation and cultural level of music students in normal colleges and universities. However, in the specific process of music education and teaching in normal universities, there are some deficiencies in the curriculum construction of music major in some normal universities. They fail to make full use of Internet information technology, pay too much attention to students' music level, and pay insufficient attention to cultural literacy, which has caused certain obstacles to the improvement of the quality of music major construction in normal universities. In addition, the status of art education of music majors in some colleges and universities is higher than that of normal education, and the music professional quality and music teaching ability of music majors in normal colleges and universities cannot be effectively improved. Therefore, in the specific process of music education in normal colleges and universities, music teachers in normal colleges and universities should further enhance their attention to students' cultural education. They should not only care about students' mastery of music knowledge and skills but also pay enough attention to and support the cultivation of students' music teaching ability, so as to ensure the teaching time of professional education and normal education. The teaching arrangement and practice content should be unified, the proportion of technical education and cultural education should be balanced, the professional informatization level should be improved, and the construction quality of music education major in normal colleges and universities and the training quality of music teachers should be improved.

RETRACTED

Because “education should aim at cultivating students' independent thinking ability and self-management ability, and provide students with the skills and abilities needed for future independent learning,” independent learning is not only necessary but also very important [1]. The so-called independent learning refers to the teaching process of students in the teacher's inspiration, guidance, and help, through their own exploration of problems, independent participation in the process of solving problems and acquiring knowledge, so as to solve problems and learn to solve problems [2]. Independent learning is a learning behavior and process that takes students as the main body of learning and realizes individual learning goals through its independent analysis, exploration, practice, questioning, and creation. With the popularity of the Internet, independent learning based on the network environment is developing rapidly [3]. Independent learning under the network environment is under the premise of making full use of network advantages, let the students with a strong desire to find problems, solve problems, and urgent mood, using the method of inquiry, independent participation in each course, so as to solve the problem, master the corresponding subject knowledge and various abilities. Independent learning as a learning method is more suitable in the network environment, because the network has a large number of resources needed for research, which helps students to establish a group cooperation mechanism, and can enable teachers to achieve asynchronous guidance [4]. At the same time, we improve the comprehensive ability of students, open up its creation.

RETRACTED

The fundamental goal of higher education is to train the innovative talents needed by the country. One of the basic laws that modern higher education must follow is to cultivate students' ability of independent learning, which is suitable for all disciplines of higher education. Music is one of the oldest and most infectious art forms of human beings. As an important form and carrier of human culture, music contains rich cultural and historical connotation, and it has a unique artistic charm. The rich cultural heritage of music art provides a very wide feasibility for students' independent study. After years of practice and exploration, the music education has accumulated some successful experience in the curriculum and teaching. However, due to the influence of the traditional teaching mode, the teaching mode and teaching method of the music education in China still follow the traditional teaching method [5]. To a large extent, teaching methods are limited to what teachers teach and what students learn, and overemphasize on the role of teachers in teaching, thus ignoring the cultivation of students' independent learning ability. Students majoring in senior teacher music have the special dual status of both current students and future teachers. If traditional education methods are used, they will directly affect the learning methods, learning attitude, knowledge structure, and skill structure of generations of educators, resulting in limitations in all aspects. In today's network environment, the independent learning of senior teacher music major students will completely overcome the limitations of traditional music education and traditional learning in space, time, education age, teaching environment, and other aspects, and meet the needs of the society to the greatest extent. The network environment provides pictures, text, sound, and similar learning signals; helps to develop innovative thinking and divergent thinking, and establish the connection between old and new knowledge; and helps students to master scientific, reasonable, and advanced learning and teaching methods, and lay a good foundation for their study and future work [6].

The curriculum construction and teaching work of music education major in normal colleges and universities need to comply with the development trend of the times; give full play to the advantages of Internet information technology, such as fast transmission speed, wide coverage, and rich information storage; and make effective use of Internet information technology in the process of music curriculum construction in normal colleges and universities. In the specific process of the teaching of music education in normal colleges and universities, the application of Internet information technology is still insufficient. First, the online communication mechanism is not perfect. Some music education majors in normal universities have not established a perfect online communication mechanism, and the communication channels between teachers and students and students are not smooth and timely, which is not conducive to the solution of students' learning problems and the improvement of teachers' teaching process. Second, the use of network music teaching resources is insufficient. Affected by the factors of not advanced equipment and low teachers' information literacy, some teachers did not make full use of information technology to collect, sort out, and use online music teaching resources, which hindered the improvement of the quality of music education courses in normal colleges and the enrichment of students' music knowledge. Finally, the innovation of teaching mode is insufficient. Some teachers have not innovated the teaching mode, but still use the traditional teaching mode. The degree of informatization of the teaching mode is not high, which has caused certain obstacles to the improvement of the music education specialty and the actual teaching quality of the curriculum in normal universities.

RETRACTED

## 2. State of the Art

At present, there is no standardized definition of learning methods, but most scholars believe that learning methods are the means and value direction to achieve learning goals. Through the analysis of the interactive learning between teachers and students, Ai Xueli (Ashley) divides the interaction into three types, namely, student center, knowledge center, and teacher center; there are different types of negotiation, noninterference, and command [7]. The concept of self-directed learning is obviously different from the types proposed above.

Scholar Professor Han Siqing (Hebei Institute of Education Science) believes that independent learning is a concept with relativity and multilevel meaning. Its relativity refers to: first, teachers' control of students and students' learning cannot completely get rid of teachers' control and pursue absolute autonomy; second, compared with “multiple control,” students' learning has its internal objective laws and independent behavior, but their learning is affected by many factors [8]. Students' autonomy in learning is not only manifested in the students' active care and role of the accumulated knowledge and experience to the society but also in the active care and role of the students' mutual relationship between various learning environments and various interactions. On schoolwork study, students should take the initiative to accept the system knowledge and experience, and attaches great importance to observation, experiment, and exploration, or teachers put forward appropriate topic, guide students through certain practical activities (both inside and outside class and social activities) to study, obviously, the meaning of students learning autonomy, and degree is also have level. Independent learning mainly includes three aspects: independent learning consciousness, independent decision making and selection ability, and self-evaluation and self-control ability after the independent completion of learning tasks [9].

RETRACTED

Scholar Pang WeiGuo professor of east China normal university thinks that for autonomous learning, it should be defined from two angles: one is from all aspects of learning, if students' learning motivation is self-driven, learning content is oneself, the choice of learning strategy is autonomous regulation, learning time is self-planning and management, students can take the initiative to build learning material and social conditions, and can make self-judgment and evaluation of learning results, and learning is autonomous [10]; another one is from the whole process of learning, if the students can determine their learning goals before learning, learning plan, in the learning of learning progress, learning methods for self-monitoring, self-regulation, after learning to self-check learning results, self-evaluation, and self-summary, and learning is autonomous [11].

To sum up, although domestic and foreign scholars have different definitions and understandings of the concept of independent learning, and have certain truth, and have formed a certain theoretical system, the core of the common point is one to improve the self-awareness of each learning subject. At present, the theory of independent study is influential in the theory is Mr. White et al. [12].

However, relatively speaking, the author thinks that there is a big gap between their definition of independent learning and the realistic independent learning, which belongs to an idealized independent learning. But the core of the common ground is to highlight the autonomous consciousness and autonomous ability of each independent learning subject. It is a kind of learning way; is a lifelong education and build learning society concept of learning way, with relative consciousness, relative independence, relatively personalized, relative effectiveness; can seek positive self-design, self-regulation, self-discovery, self-discovery, self-reflection, self-evaluation of learning strategies, and tendency. It refers to the learning activities with broad thinking and narrow concepts that give full play to the learners' self-awareness and self-ability under the guidance and encouragement of teachers [13].

RETRACTED

In addition, the development of music education and teaching in normal colleges and universities needs to make full use of Internet information technology to improve students' music level through the use of online music education resources and the Internet. Therefore, in the specific process of music education in colleges and universities, the following three aspects should be achieved. First, we establish and improve the online communication mechanism. Teachers of music education major courses in normal colleges and universities should give full play to the advantages of the Internet information technology in communication, encourage teachers and students to actively exchange existing problems and puzzles, and further improve students' understanding and mastery of music education knowledge. Second, we make full use of network music teaching resources. Teachers and students of colleges and universities should make full use of Internet teaching resources; give full play to the advantages of the high popularity of mobile network information terminals; encourage students to actively collect and sort out relevant teaching materials in their spare time, preview, and review; and constantly promote the improvement of students' learning ability. Finally, we should innovate the information-based teaching mode. Teachers should fully explore the adaptability of the information-based teaching mode to the music education courses of the university, innovate the teaching mode, improve the information-based level of the teaching mode, and promote the learning efficiency of students in normal colleges and universities.

## 3. Methodology

### 3.1. The Characteristics of Autonomous Learning

Independent learning is a process in which learners actively adjust their learning strategies and efforts according to the requirements of their own learning ability and learning tasks. Network independent learning is a new form of learning that learners use computers to surf the Internet and learn independently through the network. Its ultimate goal is to help students cultivate the ability of independent learning and the ability to effectively use various learning strategies, so as to master new knowledge independently under the condition of leaving the classroom. Through reviewing the literature, we found that learning motivation is one of the main reasons affecting students' consciousness of independent learning. Learning motivation is also the internal psychological course that causes and maintains students' learning activities and leads the learning activities to teaching [14]. It includes surface learning motivation, deep learning motivation, and target learning motivation. The surface learning motivation is that students learn music because of external motivation. Therefore, they learn only to meet the minimum standards set by teaching. These students only use mechanical memory as the main learning means in the process of music learning [15]. The deep motivation is that students have an essential and heartfelt interest in music, so they will find their own meaning in music learning. Objective learning motivation refers to a high degree of learning motivation and strong enthusiasm for learning, due to good learning habits, can arrange learning time in a planned and organized way, and try to explore the essential laws and skills of music [16].

RETRACTED

Learning motivation and learning are a dialectical relationship, learning can produce motivation, and motivation can promote learning. The effect of independent learning in the network environment depends on the choice of students' learning strategies. Among the many factors affecting the choice of learning strategies, learning motivation is one of the most important factors affecting the choice of learning strategies, which can affect students' choice of learning needs, learning consciousness, learning attitude, and learning interest [17].

In short, the characteristics of independent learning are to give full play to learners' inner potential, cultivate the habit of relatively independent learning, guide learners to develop reasonable learning goals, constantly reflect on their learning process, constantly adjust learning strategies, and constantly develop the ability of independent thinking, the ability to analyze problems, and the ability to solve problems [18].

### 3.2. Strategy Exploration of Independent Learning Motivation Activation for Students Majoring in Music Education under the Network Environment

#### 3.2.1. Establish a New Teaching Mode Based on the Classroom and the Computer Network

The basic concepts of the new curriculum standard of high normal school music are as follows: take music aesthetics as the core, cultivate interests; pay attention to music practice and enhance creative consciousness; promote folk music; and understand multicultural. As the master machine to train music teachers in primary and secondary colleges, music education majors should also follow the corresponding teaching concepts and actively cultivate innovative and comprehensive music education talents [19]. However, due to the constraints of teaching plan, teaching hours, and other aspects, there are still many deficiencies in paying attention to the development of students' personality and the cultivation of diversified culture. And based on the classroom and computer network, new teaching mode not only can emphasize classroom personalized teaching but also can fully explore students' autonomous learning ability, make the students under the guidance of teachers, according to their own characteristics, level and time, choose the right, interested in learning content, with the help of computer network, quickly improve the music comprehensive application ability, and achieve the best learning effect. The teaching model has three main components: students, teachers, and computer networks [20].

RETRACTED

On the whole, this teaching mode has the following two characteristics:

*(1) When Students Become the Main Body of Teaching Activities, They Can Adopt Personalized and Independent Learning Methods*. Under the guidance of traditional classroom methods, students are allowed to determine their learning goals, learning methods, and learning processes according to their own conditions, learning styles and learning habits; choose appropriate learning content; and, with the help of computer network resources, improve the comprehensive application ability of music to achieve the best learning effect. In some strong theoretical music courses, such as Chinese and foreign music history, teachers can, according to the different situation of students, be divided into several groups, each group of students decorates different teaching tasks: let students in extracurricular using network resources for independent learning, collect relevant learning materials, teachers in the difficulty of the next lesson on the course, make students to have a deeper understanding of interested knowledge, and can summarize. In this way, students can actively think in class, actively participate in the discussion, and gradually find their own learning goals, learning interests, and appropriate learning methods, and cultivate their own awareness of independent learning [21].

*(2) Teachers Should Change Their Roles and Build a New Teacher-Student Relationship*. In the network teaching environment, teachers must adjust the relationship between themselves and learners, and truly take the “teacher-led, students as the main body.” From the original knowledge imparting to resource developers and learning organizers, teachers guide students to carry out independent learning and cooperative learning in the classroom learning, and to help students to complete the construction of meaning in the cooperation [22].

In the choice of classroom content, teachers must change from the disseminator of knowledge to the guide and facilitator of students “learning, so as to help students learn the various knowledge, skills and strategies needed to deal with the challenges, cultivate students” metacognitive ability such as self-planning, self-regulation, and self-evaluation and improve students' independent learning level. In the control of classroom order, teachers must also change from the only controller of the classroom to the collaborator and helper of student activities; organize and supervise the interaction between students and communicate between teachers and students; and constantly encourage students, so that students are full of hope for music learning. And from a single “professional” teachers to “compound” learning researchers, teachers in addition to have professional knowledge and skills and related pedagogy, psychology knowledge, also must master the method of using network technology and basic music software operation skills, and summarize the accumulated experience, to form the understanding of regularity. In this way, as a professional institution of higher learning training, a new generation of teachers, in addition to use oral language and blackboard to impart knowledge information, also good at network-rich network resources, using a variety of information carrier, to scientific, accurate, image, vivid impart knowledge, and transfer all kinds of information, further establishes a new teaching mode based on classroom and computer network [23].

RETRACTED

#### 3.2.2. Set Reasonable Learning Goals

The establishment of learning goals means the establishment of a standard of struggle, an intention to obtain some kind of success in learning. Through this standard and intention throughout the subsequent daily life, it can provide learners with strategies to realize their dreams and goals, avoid students' aimless and directional learning, and realize their life value to the maximum extent [24].

The development of reasonable learning goals for students majoring in music education should be completed with the guidance and help of teachers. Teachers can help them to set their learning goals as both general goals and special goals. The realization of general goals has long-term characteristics, which can be “study hard during college, further study after graduation,” “strive for good results,” “to be an excellent student,” and other goals. Special goals are clear and specific, such as “write a study feeling every week,” “listen to a music work every day,” and other short-term goals, the general goals need to be implemented through the realization of special goals [25].

For the formulation of special goals, teachers can inform the learning plan of the course at the beginning of the semester course and assign students some after-class thinking questions in each class so that students can acquire knowledge through the network and other means, so as to complete the construction of their own knowledge, stimulate the deep learning motivation, and achieve the expected learning goals.

RETRACTED

As for setting general goals, teachers must find out students' unique needs and interests through surveys and individual interviews to help them determine their individual goals. For example, teachers can according to the different characteristics of each student, explore each student's own strengths and advantages, and guide them to establish the idea of subject learning, university learning idea, after graduation life planning, etc. Only under the guidance and help of teachers, students according to their own situation, and strive to implement, can greatly stimulate students' deep learning motivation, improve their interest in learning, to achieve the predetermined personal goals.

### 3.3. Optimize the Artistic Value Orientation of Music Major in Normal Universities

The development of curriculum construction and teaching work of music education major in normal colleges and universities is an innovation and improvement of the construction of music education major in normal colleges and universities on the basis of traditional music education. Therefore, the following three aspects should be achieved in the specific construction of music education major and the development of teaching work in normal colleges and universities. First, we carry out aesthetic education. Teachers should pay more attention to students' artistic cultivation and music appreciation ability, and carry out aesthetic education to create an aesthetic atmosphere for students and improve their art appreciation ability. Second, we pay attention to artistic cultivation. Teachers need to pay more attention to students' music perception ability and their inner world, actively guide and guide students' problems, avoid students' utilitarian tendency in the course of music education curriculum construction, help students establish correct professional ethics and values, and promote the improvement and all-round development of students' professional quality. Finally, we improve the teaching evaluation indicators. Leaders and teachers of normal colleges and universities should further optimize the evaluation mode, combine process evaluation with result evaluation, encourage students to adjust their learning plans and learning methods, guide students to correct their learning attitude, change the one-sided concept of paying too much attention to examination results, and promote the improvement of students' music level and artistic accomplishment.

RETRACTED

## 4. Result Analysis and Discussion

### 4.1. Analysis of the Current Situation of Music Learning Methods

The main purpose of the survey is to carry out the corresponding problems of the high music course teaching link and understand the students' music course learning way. Through multiple aspects of the analysis of the higher teacher training colleges, music teaching situation, on the basis of the survey status of relevant suggestions, hopes to help the future music teaching mode change reference, which contributes to the music teaching field in our country.

In order to further ensure the feasibility of the questionnaire, a preliminary test was carried out before issuing the questionnaire, selecting 50 students in the higher teacher training colleges for the preliminary survey, recycling the questionnaire, and carrying out preliminary verification. The reliability coefficient was analyzed by SPSS software, and the main index is a reliability coefficient. From 0.8 to 0.9, the reliability is good; between 0.7 and 0.8 and 0.65∼0.7, the questionnaire should be adjusted again. Combined with the preliminary survey results of this survey, corresponding a coefficient of each dimension of the questionnaire is 0.8. The above has verified that the temperature questionnaire is good. In addition, in order to analyze the validity of the questionnaire, a further KMO test was also carried out. The result was 0.870, indicating that the questionnaire had good validity. Later, a formal survey was carried out, and a total of 350 questionnaires were issued, and 325 were recovered, with a recovery rate of 92.8%.

This survey is mainly in the aspect of classroom students' independent experience. According to the survey results, the specific content of the classroom independent learning experience is as shown in Figure 1.

Through the survey and analysis of “in the music class,” we can learn that 47% of students noticed “occasionally”; 14% said “often” and 32% said “no.” as shown in Figure 2.

Through the survey and analysis of “did the teacher let the students create music or show their understanding of music on stage,” we can understand that 39% said “occasional” attention; 21% said “often” and 40% said “no” as shown in Table 1.

It can be seen from Table 1, in music classroom learning, the most popular among students is “learning to sing,” followed by “music activities” and “appreciating famous music.” The classroom music teaching least popular by students is “music theory knowledge,” which may be related to the relatively boring music theory knowledge and students' low interest in learning. The more interested students are in the classroom practice, the stronger the experience it will bring to students. Teachers should pay attention to this and carry out more classroom music teaching that students are interested in so that students can better conduct experiential learning.

RETRACTED

According to the above survey results, in the process of students' experience learning, occasionally, and not accounted for a large proportion, while the students' experience in the music class was low. In this case, teachers may lack of trust in students in the process of music classroom teaching. In the process of regulating students, flexible measures will lead to too loose classroom discipline management, which leads to poor classroom discipline, affecting the actual effect of high normal school music teaching and students' no sense of participation and experience. So, the teacher should pay attention to the students' experience and emphasize the students' active participation in the music class, it is necessary to stimulate students in music form and music emotional positive experience of association and imagination, the new curriculum also emphasizes the students' aesthetic experience process and emphasizes the value of the music teaching process itself; then, the music classroom will present the dynamic interaction between teachers. Student content and environment thus get rid of simple music learning based on knowledge transfer and skill training, and turning to situational learning of behavioral experience.

### 4.2. Survey and Analysis of Students' Independent Music Study

The purpose of this survey is to understand the students' interest in music courses, their corresponding abilities, and the active and passive reactions reflected in music learning. The details are shown in Table 2.

To understand students' initiative in music learning, this paper does a survey as shown in Table 3, most of the students are more active and active, more than half of the students can carry out active learning, a few students play only under the supervision of the students' parents, and teachers can better carry out learning.

Using any music from teachers in other subjects, 55% reported “occasional” attention, 23% reported “frequent,” and 22% reported “no” as shown in Figure 3.

According to the survey and analysis of whether they have any interest in learning music after class, we can understand that 47% of students said “occasionally,” 21% said “regular,” and 32% said “no” as shown in Figure 4.

According to the survey “have you heard any course or lecture on music on the Internet,” 40% said “occasionally,” 18% “regular,” and 42% “no” as shown in Figure 5.

RETRACTED

According to the above survey results, in the process of students' independent learning, they occasionally do not account for a large proportion, and their interest in independent music learning is weak, most of which belong to passive learning. In this case, passive learning means that students rely too dependent on teachers or others for music learning. During the process of music learning, the objectives, contents, and processes of music learning are determined by the teacher or others. Students have no self-plan and a lack of internal motivation. Obviously, self-learning is a high-quality learning method when compared to passive learning. Therefore, music learning should abandon passive learning methods and choose independent learning methods that can reflect initiative. In music, which is still not the focus of high normal school entrance examinations, interests and hobbies are the main drivers of music learning. Relying on students' interest in learning, self-study is in higher teacher training colleges. For those students who are not very interested in music, they can find their interest points in the network information. In view of the diversified music situation and the continuous innovation and development of music, teachers should actively use students' preferences to guide them to realize the integration of online and offline so that students can achieve the transformation from passive learning to independent learning.

### 4.3. Investigation and Analysis of Students' Inquiry Study of Music

The survey is mainly to understand whether students have actively explored and thought deeply about music, as well as the learning and communication with music teachers in music. The details are shown in Table 4.

Through the “you know the form of inquiry learning” survey data analysis, we can see the table to understand: more than 70% of the students can independent cooperation and explore, and have a certain understanding of independent inquiry and cooperation to explore this form overall relatively low; more than half of the students have a certain degree of understanding and, at the same time, have nearly 20% of the students who understand the corresponding principle; and only a few students do not understand this content. On the whole, most of the students have a certain degree of understanding of inquiry learning, and the most familiar type of learning is independent inquiry, followed by cooperative inquiry, which may be closely related to the type of teacher activities, and may also be related to the hardware facilities provided by the school.

Through the survey and analysis of the music in the process of listening to music, we can understand that 48% noticed “occasionally,” 24% said “often,” and 28% said “no” as shown in Figure 6.

RETRACTED

From the above survey results, in the process of students' learning and exploration, occasionally and not a large proportion, the music exploration and communication with teachers are rare. In this case, students should be encouraged to explore themselves, group cooperation, ask questions, collect information, and complete the query process through communication. Compared with inquiry learning, acceptance learning is mainly through teacher teaching or demonstration, as well as students' listening or watching. The content of music learning is presented in a clear way.

## 5. Conclusion

We establish appropriate independent learning objectives to enhance students' motivation and learning fun; develop effective independent learning plan to further standardize student learning and achieve goals quickly; use good learning strategies, answer questions; guide students to use the network reasonably, continuously strengthen self-protection consciousness; and teach students to learn self-evaluation and accumulate learning experience. To sum up, only then, the students can better carry out autonomous learning in the network environment.

Although the research of independent music learning has formed a certain situation, the systematic research based on independent learning of higher vocational music in China is still lagging behind. Therefore, many aspects of this topic in the field of independent higher vocational music learning and research are only made superficial exploration, which is the so-called stone to ask the way, and cross the river by feeling the stone. For example, ① it has a weak research on independent evaluation mechanism and offers some opinions, but still far from the practical operation; ② it combines independent learning classroom with extracurricular teaching activities enough; ③ it supports the rationality of music aesthetics, music philosophy, and music psychology. In the future, we can try to combine the independent evaluation mechanism mentioned in this paper and the goal of combining independent learning classroom with extracurricular teaching activities through offline ways.

## Figures and Tables

**Figure 1:** The teacher lets the students feel the music in the music class.

**Figure 2:** The teacher lets the students feel the music in the music class.

**Figure 3:** Music played to the teachers during the learning process.

**Figure 4:** Interest in learning music after class.

**Figure 5:** Listening to courses or lectures about music on the Internet.

**Figure 6:** An in-depth analysis of the music.

**Table 1:** Students' favorite music learning experience.

Choice	Knowledge of music theory (%)	Appreciate famous song (%)	To compile a musical composition (%)	Learn to sing (%)	Music activity (%)
Proportion	11.32	38.49	23.89	73.67	51.76

RETRACTED

**Table 2:** Students' understanding of music learning objectives.

Choice	Be confident and know your goals clearly (%)	Sometimes I forget my goals. Sometimes I forget my goals (%)	I think a lot, but I do not know how to do it (%)	There is no goal at all (%)
Proportion	31.27	41.73	23.33	3.67

Based on the above survey, 31% shows that the students are more aware of the goals of music courses and how to develop later. Four percent of the students had no learning goals at all, and even understood the learning goals, which would have a certain impact on the analysis of the investigation. Overall, students choose the highest proportion of “sometimes forget their goals” and still have unclear goals for music learning.

**Table 3:** Students take the initiative to learn music when there is no supervision from parents and teachers.

Choice	Be able to learn actively (%)	Sometimes I take the initiative to learn not to control myself, but also forget (%)	I cannot control myself. I just want to play or rest (%)	Never take the initiative to learn (%)
Proportion	43.12	54.55	2.33	0.00

**Table 4:** Students' knowledge of the form of inquiry learning.

Choice	Independent inquiry (%)	Cooperative research (%)	Probe into the problem (%)	A probe into the theory of music (%)	I do not know (%)
Proportion	76.44	75.04	42.67	19.03	6.66

## Data Availability

The labeled dataset used to support the findings of this study is available from the author upon request.
